The article "Evaluation of Pulsed Electromagnetic Field Effects: A Systematic Review and Meta-Analysis on Highlights of Two Decades of Research In Vitro Studies" was published in 2021. Journal: Biomed Res Int.

# Evaluation of Pulsed Electromagnetic Field Effects: A Systematic Review and Meta-Analysis on Highlights of Two Decades of Research In Vitro Studies

**DOI:** 10.1155/2021/6647497

**Published:** 2021-07-29

**Authors:** Mahsa Mansourian, Ahmad Shanei

**Affiliations:** ^1^Department of Medical Physics, Faculty of Medicine, Isfahan University of Medical Science, Isfahan, Hezar Jerib Avenue, Isfahan, Iran; ^2^Department of Medical Physics, Faculty of Medical Science, Isfahan University of Medical Science, Isfahan, Hezar Jerib Street, Isfahan, Iran

## Abstract

Pulsed electromagnetic field (PEMF) therapy is a type of physical stimulation that affects biological systems by producing interfering or coherent fields. Given that cell types are significantly distinct, which represents an important factor in stimulation, and that PEMFs can have different effects in terms of frequency and intensity, time of exposure, and waveform. This study is aimed at investigating if distinct positive and negative responses would correspond to specific characteristics of cells, frequency and flux density, time of exposure, and waveform. Necessary data were abstracted from the experimental observations of cell-based in vitro models. The observations were obtained from 92 publications between the years 1999 and 2019, which are available on PubMed and Web of Science databases. From each of the included studies, type of cells, pulse frequency of exposure, exposure flux density, and assayed cell responses were extracted. According to the obtained data, most of the experiments were carried out on human cells, and out of 2421 human cell experiments, cell changes were observed only in 51.05% of the data. In addition, the results pointed out the potential effects of PEMFs on some human cell types such as MG-63 human osteosarcoma cells (*p* value < 0.001) and bone marrow mesenchymal stem cells. However, human osteogenic sarcoma SaOS-2 (*p* < 0.001) and human adipose-derived mesenchymal stem cells (AD-MSCs) showed less sensitivity to PEMFs. Nevertheless, the evidence suggests that frequencies higher than 100 Hz, flux densities between 1 and 10 mT, and chronic exposure more than 10 days would be more effective in establishing a cellular response. This study successfully reported useful information about the role of cell type and signal characteristic parameters, which were of high importance for targeted therapies using PEMFs. Our findings would provide a deeper understanding about the effect of PEMFs in vitro, which could be useful as a reference for many in vivo experiments or preclinical trials.

## 1. Introduction

Electromagnetic fields (EMFs) are composed of magnetic and electric fields that influence each other [1]. There are many EMF subtypes with varying frequency rates, and they can cause either positive or detrimental biological effects. For medical purposes, they can be used in diagnostic modality and be considered as a potential therapeutic option as well. On the other hand, EMFs can penetrate tissues without experiencing intensity decrement [2], pass through the cell membrane, and affect cell responses. Consequently, cells may experience diverse pathophysiological disorders like cancer, thus, elevating one's concern during the course of using EMFs for therapeutic purposes [3]. However, despite many findings, the carcinogenic role of EMF is still unclear.

The article "Evaluation of Pulsed Electromagnetic Field Effects: A Systematic Review and Meta-Analysis on Highlights of Two Decades of Research In Vitro Studies" was published in 2021. Journal: Biomed Res Int.

Among subtypes of EMFs, low-frequency fields with specific amplitudes and waveforms are referred to as pulsed EMFs (PEMFs) [4]. Being a promising strategy and a type of the noninvasive and inexpensive physical approaches, PEMFs have exhibited therapeutic potential for treating various diseases [5]. It has already been shown that they can make changes to cell cycle, apoptosis, cell proliferation, and differentiation. Indeed, they are able to affect and alter the cell function by inducing forced vibration for free ions on the cell membrane surfaces due to an external oscillating field [6]. Irregular gating of ion channels triggered by this situation can certainly disturb the balance of transmembrane proteins and, consequently, disrupt cell function [7]. It has also been proposed that the effect of PEMFs may be propagated and amplified along the whole signal transduction pathway, thereby changing cell behavior [8]. In some studies, it has been reported that PEMFs can modulate both downstream signal transduction pathway and cell surface receptor expression/activation [8, 9]. As a result, homeostatic cell functions such as differentiation, viability, proliferation, interaction with components of extracellular matrix (ECM), and communication with neighboring cells could be restored [10]. In addition, PEMFs could enhance both the neurogenic differentiation of mesenchymal stem cells (MSCs) and osteogenic differentiation. Because EMFs easily permeate through cells [4] and change the electric field of the inner cell membrane, they can induce biological changes. In particular, they can induce changes in the Ca^2+^ efflux and, consequently, modulate various biological effects such as nitric oxide signaling, growth factor secretion, and Mitogen-Activated Protein Kinase (MAPK)/Extracellular Signal-Regulated Kinase (ERK) [11]. It has been hypothesized that the production of second messengers is stimulated by the direct effect of PEMF on phospholipids within the plasma membrane, and subsequently, multiple intracellular signal transduction pathways are initiated [12].

The article "Evaluation of Pulsed Electromagnetic Field Effects: A Systematic Review and Meta-Analysis on Highlights of Two Decades of Research In Vitro Studies" was published in 2021. Journal: Biomed Res Int.

There are many factors affecting the biological responses. To clarify PEMF impacts, studies have reported that signal characteristics play a crucial role in determining the type of biological responses including amplitude and frequency of exposure to the applied PEMF [13]. Indeed, to deliver a therapeutic PEMF, it is necessary to optimize these important parameters [6]. In addition, a large volume of evidence has revealed that some kinds of cells appear exquisitely sensitive to PEMF, while other types appear relatively unresponsive. For instance, undifferentiated PC12 cells are more sensitive to PEMF exposure, while differentiated PC12 cells are more resistant to stress [14]. Consequently, cell properties are of vital importance in establishing a biological response to PEMF in vitro.

Despite a relatively long history of using PEMFs in medicine, little is known about the biological mechanism of such therapies. To develop a reliable working principle of PEMF therapies, it is worth investigating the experimentally observed biological effects caused by these fields alone. Thus, in this study, a meta-analysis was performed using 3249 in vitro experimental observations available in 92 scientific journals (1999-2019) in order to determine the potential effects of PEMF on different cell types of both human and rat/mouse. Our analysis scrutinized the published experiments that had considered the effects of exposure to PEMFs (cytogenetic, gene, and protein expression analysis) on cell types from rats, mice, and humans to gain a more explicit and evidence-based conclusion on the association between PEMFs and cell responses.

## 2. Material and Methods

In Tables 1–15, the characteristics of experimental protocols and variables are presented. In this paper, cellular response (presence or absence) in human, mouse, or rat cells is defined as changes due to exposure to PEMFs. We analyzed the reported studies based on the different experimental readouts/endpoints which they used for their studies and the physiological variables they measured. These studies are shown in Figures 1–3, (human cells), Figure 4 (rat/mouse cells), and Figure 5 (other species), separately.

### 2.1. Collection of Raw Data

An electronic literature search of databases including Web of Sciences and PubMed was conducted for publications in English from 1999 up to 2019. The key terms introduced in the search engines included “pulsed electromagnetic fields” and “cell.” The process of selecting the papers was carried out by reading the titles and abstracts of the studies as well as the full article when necessary. Upon omitting duplicate titles, full-text versions of the selected papers were obtained.

The article "Evaluation of Pulsed Electromagnetic Field Effects: A Systematic Review and Meta-Analysis on Highlights of Two Decades of Research In Vitro Studies" was published in 2021. Journal: Biomed Res Int.

We excluded those experiments that (1) targeted direct animal or human exposure followed by the analysis of individual cells and (2) applied the combination of PEMFs and other effective treatments, e.g., chemotherapy. After screening many research studies, 92 papers with different designs were eligible for meta-analysis.

For data analysis, the cell responses were classified as “presence” (PEMF exposure changed the cell response statistically significantly in comparison to the control group regardless of direction) and “absence” (no significant PEMF effect).

For each included study, the following data were extracted: type of cells, pulse frequency of exposure, exposure flux density, time of exposure, waveform, and assayed cell responses (cells, cell function, and DNA). Bibliographic details of the studies including the first author and year of publication were also retrieved.

### 2.2. Analysis of Raw Data

According to the above explanations, given that the frequency and intensity of the mentioned exposure differ across studies, achieving different biological responses would not be unexpected. In this respect, we pooled the retrieved experimental data based on used pulse frequencies and flux densities. Our analysis considered the effect of several subgroups of pulse frequency and flux density as follows: (a) 0.1 < *ƒ* ≤ 10 Hz, (b) 10 < *ƒ* ≤ 100 Hz, (c) 100 < *ƒ* Hz, (d) *I* < 1 mT, (e) 1 ≤ *I* < 10 mT, (f) 10 ≤ *I* < 100 mT, and (g) 100 mT ≤ *I*. Also, subgroups of exposure time and waveform were considered as follows: (H) acute exposure ≤ 24 h, (I) acute exposure > 24 h, (J) chronic exposure ≤ 10 days, (K) chronic exposure > 10 days, (L) square wave, (M) the bursts consisted of a series of consecutive, (N) triangle wave, and (O) other waveforms.

### 2.3. Statistical Analysis

Microsoft Excel was used to organize the initial data and build a database. Meta-analysis combined the results obtained from separate studies with a similar outcome. The pooled results were obtained based on cell type, frequency, and intensity. A random-effect model was used to facilitate conducting the analysis, through which *I*^2^ value was calculated as the indicator of heterogeneity. *I*^2^ values greater than 50% could imply significant heterogeneity between the related studies. Also, the random-effect model could account for the above variation between studies, and thus, it achieved more conservative results than a fixed-effect model. Sensitivity analysis was performed to determine the effect of a particular study on the overall effect size. The presence of publication bias was tested using Begg's and Egger's regression asymmetry tests [9]. Statistical analyses were conducted using STATA version 14.0. A *p* value less than 0.05 was considered significant for all tests.

The article "Evaluation of Pulsed Electromagnetic Field Effects: A Systematic Review and Meta-Analysis on Highlights of Two Decades of Research In Vitro Studies" was published in 2021. Journal: Biomed Res Int.

## 3. Results

A number of publications are analyzed in Figure 6, which provides an overview of the years of publication. Cellular response (presence or absence) was observed in human cells (2441 experiments in Figures 1–3), rat or mouse cells (854 experiments in Figure 4), and other species (11 experiments in Figure 5). The results indicated that most of the experiments were carried out on human cells, among which stem cells drew greater experimental attention. Of not, in case the analysis incorporated such parameters as exposure to PEMFs and individual cell types, the potential effects of PEMFs on cell types, such as bone marrow mesenchymal stem cells (BM-MSCs) (based on 559 reported experiments, *p* value < 0.001), would become clear. However, based on the reported evidence, no such effect was observed for human adipose-derived mesenchymal stem cells (AD-MSCs) and human osteogenic sarcoma SaOS-2 (*p* < 0.001). As a result, despite the higher susceptibility of cancer cells to PEMFS than that of other cell types, various cancer cells respond differently to PEMF stimulation.

We categorized different experimental techniques as follows: (a) cell structure (cell viability, cell morphology, apoptosis, cell proliferation, and cell differentiation), (b) cell functions (calcium concentration, signal transductions, enzyme activity, membrane potential, and membrane stability), and (c) DNA (gene expression, protein expression, ROS production, chromosome aberration, micronucleus assay, DNA damage, oxidative stress, DNA single-strand breaks, DNA double-strand breaks, and genotoxicity) in Figure 7. Our analysis of the reported results (Figure 8) suggests that most of the experiments used experimental techniques for DNA including gene expression, protein expression, and ROS production for assaying the effect of PEMFs on cells.

We also considered the effects of different pulse frequencies of PEMFs and intensity. To do so, we pooled experimental data based on the frequencies (Figure 9), intensity levels (Figure 10), time of exposure (Figure 11), and waveforms (Figure 12) used in each experiment of the 92 publications Among subgroups of frequencies, significant effects were observed at 100 Hz < *ƒ* (*p* < 0.001). However, at frequencies smaller than or equal to 10 Hz, no statistically significant effects were observed. Among subgroups of intensities, the presence of response as a result of PEMFs was seen significantly in intensities between 1 and 10 mT (*p* < 0.05) Analysis of different times of exposure in the studies indicated on effectiveness of PEMFs in chronic exposure > 10 days (*p* < 0.001) and absence of cell response in acute exposure > 24 h (*p* < 0.001).

The article "Evaluation of Pulsed Electromagnetic Field Effects: A Systematic Review and Meta-Analysis on Highlights of Two Decades of Research In Vitro Studies" was published in 2021. Journal: Biomed Res Int.

The cells exposed to PEMFs in in vitro experiments, which reported results (cellular response, either presence, or absence Table 1) under different exposure conditions, are shown as follows: (a) classification of experimental techniques in Figure 8, (b) frequency of PEMFs in Figure 13, (c) intensity levels in Figure 14, (d) time of exposure in Figure 15, and (e) waveform in Figure 16. It should be noted that our statistical test only reports the presence or absence of cellular responses in the literature, and it is not concerned with the increased or reduced effect of the mentioned responses.

## 4. Publication Bias and Sensitivity Analysis

The results of Egger's and Begg's test demonstrated no publication bias in the meta-analysis of cellular response (presence or absence) in human cells, rat or mouse cells, and other species according to different frequencies and intensity levels (*p* values for Begg's test and Egger's test for all categorizes were >0.05). To evaluate the effect of each single study on the pooled effect size, we removed each study, one by one. We found no significant effects of any individual study on the combined effect sizes in different meta-analysis presentation.

## 5. Discussion

This study scrutinized the related scientific literature for the association between PEMFs and cell responses in vitro. Realizing that there were distinctions between cell types in terms of apoptosis, rate of proliferation and age, and other characteristics and that PEMFs parameters can be characterized in terms of frequency, intensity, time of exposure, and waveform, we investigated if there were distinct properties of positive and negative findings associated with these characteristics. The results showed that there was no significant difference between the presence and absence of the cell response to PEMF stimulation in human cells, rat/mouse cells, and other species (Figure 17 for each row (*p* > 0.05)). However, several aspects of our results are notable, which are given below.

Our findings demonstrated that in in vitro studies, nearly 50% of human cells (Figure 17) would undergo changes due to PEMFs, whereas fewer number of cells in rats/mice (44.61%) and other species (18.18%) were influenced by PEMFs. Thus, a large number of experiments on cells in rats/mice and other species pointed out the absence of any effect caused by PEMFs. Among the studies conducted on human cells, most of them were performed on stem cells. According to the results, it seems that the type of stem cell plays as an effective factor in intracellular processes affected by PEMFs. Especially, in the field of bone tissue engineering in which mesenchymal stem cells are activated by EMF, this finding would be considerable.

The article "Evaluation of Pulsed Electromagnetic Field Effects: A Systematic Review and Meta-Analysis on Highlights of Two Decades of Research In Vitro Studies" was published in 2021. Journal: Biomed Res Int.

Another significant finding of our study was among osteoblast-like cells, MG-63 human osteosarcoma cells seem to be very sensitive to PEMFs (86.1%). The studies have shown that these fields could alter activity through changes in local factor production [4]. However, in human osteogenic sarcoma SaOS-2, the absence of cell response to PEMFs alone was greater in degree than the presence of cell response (75%). PEMFs appeared to have little effect on the phenotype and number of SaOS-2 cells [7].

The potential effects of PEMFs on tendon cells showed that these fields (87.74%), focusing on the potential applicability of this cell source for regenerative medicine purpose, could be effective in the treatment of tendon disorders. In fact, these fields could influence the proliferation, release of anti-inflammatory cytokines, tendon-specific marker expression, and angiogenic factor in healthy human TCs culture models [15].

Analysis of the results of other related studies concerning the effect of PEMFs on the cells of blood cancers like leukemia and lymphoma in human (and on basophilic leukemia cells in rats/mice) showed that these cells were not affected to PEMFs. Thus, it seems that these fields alone are not an effective treatment for blood cancers. Further investigations are required to examine the responsiveness of different types of blood cancer cells to PEMFs. Evaluation of different experimental techniques used in the studies showed that most of the experiments were carried out on the expression of genes and proteins, because PEMFs could verifiably promote bone fracture healing and enhance the maturation of osteoblastic cells. Also, most of studies have examined the effect of osteogenic differentiation of these fields on mRNA level.

Another part of this study focused on evaluating the role of intensity and frequency of PEMFs in stimulating cellular responses in the subgroups. This research was subject to some constraints; first, some of the related experimental studies did not provide sufficient descriptions of exposure signal characteristics, especially in expressing waveform, which in turn made us unable to interpret the results fully. Nevertheless, analysis of frequencies of PEMFs used in the studies showed that different frequencies corresponded to different levels of cellular response. In the subgroups, frequencies higher than 100 Hz and intensities between 1 and 10 mT seemed to be more effective in establishing a cellular response. In addition, the analysis of times of exposure showed that in chronic exposure to PEMF more than 10 days may observe the effect of these fields (presence: 57.66%, absence: 42.34%; *p* < 0.01), while acute exposure more than 24 h may cause to less effect (presence: 17.87%, absence: 82.13%, *p* < 0.01).

The article "Evaluation of Pulsed Electromagnetic Field Effects: A Systematic Review and Meta-Analysis on Highlights of Two Decades of Research In Vitro Studies" was published in 2021. Journal: Biomed Res Int.

It is worth noting that we may be able to find optimal parameters of PEMF in future studies in the effective ranges obtained from the present study to achieve the most effective response, depending on the desired effect.

Basically, in vitro studies use cells to investigate the interaction mechanisms better by breaking down the complexity of a whole organism into a controllable system. Indeed, each cell with a model system of its own could be suitable for a specific biological aspect. Therefore, although it cannot be expected that humans respond to PEMFs, studies of simple biological systems can advance our understanding about which systems in the body are more susceptible to PEMFs. Therefore, conducting an analysis similar to the present meta-analysis could be useful as a reference for many epidemiological studies or in vivo experiments using the whole organism animal models.

## 6. Conclusion

To the best of our knowledge, no other meta-analysis has investigated the effects of PEMF on cell responses in vitro. The findings of this study provided us insight into that which cell types could be more responsive to PEMFs. Additionally, we determined the range of frequencies and intensities which PEMFs appeared more effective. Future research would need to explore the effects of other variables on cell response in vitro and to investigate the effectiveness of PEMFs in vivo.

## Figures and Tables

**Figure 1:** Human cells (stem cells): cellular response (presence or absence) for cultured human cells (3249 in vitro exposures) pooling data from 92 peer-reviewed scientific articles published in 1999-2019. Statistical significant cell groups are highlighted. Heterogeneity results: *I*^2^ = 92.03, *p* value < 0.001.

**Figure 2:** Human cells (cancer cells): cellular response (presence or absence) for cultured human cells (3249 in vitro exposures) pooling data from 92 peer-reviewed scientific articles published in 1999-2019. Statistical significant cell groups are highlighted.

**Figure 3:** Human cells (other normal cells): cellular response (presence or absence) for cultured human cells (3249 in vitro exposures) pooling data from 92 peer-reviewed scientific articles published in 1999-2019. Statistical significant cell groups are highlighted. Heterogeneity results: *I*^2^ = 92.03, *p* value < 0.001.

**Figure 4:** Rat/mouse cells: cellular response (presence or absence) for cultured rat/mouse cells (3249 in vitro experiments) pooling data from 92 peer-reviewed scientific articles published in 1999-2019. Statistical significant cell groups are highlighted. Heterogeneity results: *I*^2^ = 56.25, *p* value < 0.001.

The article "Evaluation of Pulsed Electromagnetic Field Effects: A Systematic Review and Meta-Analysis on Highlights of Two Decades of Research In Vitro Studies" was published in 2021. Journal: Biomed Res Int.

**Figure 5:** Other species cells: cellular response (presence or absence) for cultured species cells (3249 in vitro experiments) pooling data from 92 peer-reviewed scientific articles published in 1999-2019. Heterogeneity results: *I*^2^ = 70.90, *p* value = 0.064.

**Figure 6:** Overview of the published year: cellular response (presence or absence) for cultured human, rat/mouse, and other species cells (3249 in vitro exposures) pooling data from 92 peer-reviewed scientific articles. Heterogeneity results: *I*^2^ = 36.12, *p* value = 0.049.

**Figure 7:** Different experimental techniques: cellular response (presence or absence) for cultured human, rat/mouse, and other species cells (3249 in vitro experiments) pooling data from 92 peer-reviewed scientific articles. Heterogeneity results: *I*^2^ = 98.49, *p* value < 0.001.

**Figure 8:** Classification of experimental techniques observed from 3306 experiments from 92 peer-reviewed scientific publications (1999-2019). Cells exposed to PEMFs in vitro experiments that reported results (cellular response (presence or absence)) for different exposure conditions (frequency and intensity). These experimental techniques are classified as (i) cells (cell proliferation, cell differentiation, cell viability, cell morphology, and apoptosis), (ii) cell functions (enzyme activity, calcium concentration, signal transductions, membrane potential, and membrane stability), and (iii) DNA (chromosome aberration, micronucleus assay, DNA damage, oxidative stress, DNA single-strand breaks, DNA double-strand breaks, genotoxicity, gene expression, protein expression, and ROS production).

**Figure 9:** Different frequency levels: cellular response (presence or absence) for cultured human, rat/mouse, and other species cells (3249 in vitro experiments) pooling data from 92 peer-reviewed scientific articles published in 1999-2019. Please note that frequency values were not given in 85 experiments/exposures. Heterogeneity results: *I*^2^ = 96.7, *p* value < 0.001.

**Figure 10:** Different intensity levels: cellular response (presence or absence) for cultured human, rat/mouse, and other species cells (3249 in vitro experiments) pooling data from 92 peer-reviewed scientific articles published in 1999-2019. Please note that intensity values were not given in 624 experiments/exposures. Heterogeneity results: *I*^2^ = 92.36, *p* value < 0.001.

**Figure 11:** Different time of exposure: cellular response (presence or absence) for cultured human, rat/mouse, and other species cells (3249 in vitro experiments) pooling data from 92 peer-reviewed scientific articles published in 1999-2019. Please note that intensity values were not given in 624 experiments/exposures. (a) Heterogeneity results: *I*^2^ = 0.3, *p* value = 0.765.

The article "Evaluation of Pulsed Electromagnetic Field Effects: A Systematic Review and Meta-Analysis on Highlights of Two Decades of Research In Vitro Studies" was published in 2021. Journal: Biomed Res Int.

**Figure 12:** Different waveforms: cellular response (presence or absence) for cultured human, rat/mouse, and other species cells (3249 in vitro experiments) pooling data from 92 peer-reviewed scientific articles published in 1999-2019. Please note that intensity values were not given in 624 experiments/exposures. (b) Heterogeneity results: *I*^2^ = 0.45, *p* value = 0.87.

**Figure 13:** Frequency range observed from 3306 experiments studies from 92 peer-reviewed scientific publications (1999-2019). Cells exposed to PEMFs in vitro experiments that reported results (cellular response (presence or absence)) for different exposure conditions (frequency and intensity). Frequency values are shown in Hz.

**Figure 14:** Intensity observed from 3306 experiments from 92 peer-reviewed scientific publications (1999-2019). Cells exposed to PEMFs in vitro experiments that reported results (cellular response (presence or absence)) for different exposure conditions. Intensity values are shown in mT.

**Figure 15:** Time of exposure observed from 3306 experiments from 92 peer-reviewed scientific publications (1999-2019). Cells exposed to PEMFs in vitro experiments that reported results (cellular response (presence or absence)) for different exposure conditions.

**Figure 16:** Waveforms observed from 3306 experiments from 92 peer-reviewed scientific publications (1999-2019). Cells exposed to PEMFs in vitro experiments that reported results (cellular response (presence or absence)) for different exposure conditions.

**Figure 17:** Cellular response (presence or absence) for cultured human, rat/mouse, and other species cells (3249 in vitro exposures) pooling data from 92 peer-reviewed scientific articles published in 1999-2019. Heterogeneity results: *I*^2^ = 88.92, *p* value < 0.001.

**Table 1:** Statistically significant difference cell groups from Figures 1–3.

Exposure detail	Total	Studies with statistical significant cellular response	
		Presence	Absence
Human	14	3 (21.43%)	11 (78.57%)
Rat/mouse	5	2 (40%)	3 (60%)
Other species	0	0	0

Total cells	19	5 (23.81%)	14 (76.19%)

**Table 2:** Human cell studies: PEMFs exposure conditions used in in vitro studies.

No.	Cell line	Frequencies and intensities	Cell response	Result	Year	First author
1	Retinal pigment epithelial (RPE) cells	Frequency of 50 Hz Intensity of 1 mT	Cell proliferation, cell death, and gene expression	Transcript levels of proangiogenic genes (HIF-1*α*, VEGFA, VEGFR-2, CTGF, cathepsin D TIMP-1, E2F3, MMP-2, and MMP-9) increased	2019	Oladnabi et al. [56]
2	Adipose-derived mesenchymal stem cells (AD-MSCs)	Frequency of 5 Hz Intensity of 1.1 mT	Cell proliferation	PEMF can be beneficial to tissue-derived stem cell proliferation	2018	Daish et al. [16]
3	Adipose-derived stem cells (ASCs)	Frequency of 50 Hz Intensity of 1 mT	Cell proliferation, cell differentiation Gene expression Protein expression	PEMF could promote cell proliferation and osteogenic differentiation. Bone-related gene expression and protein expression of OPN, OCN, and RUNX-2 increased	2018	Yin et al. [17]
4	Human adipose-derived mesenchymal stromal cells (hAMSC)	Frequencies:10, 16, 20.6, 23.8, 26, 33, 49.9, 52.3, 75.6, and 90.6 Hz	Cell proliferation, gene expression Protein expression	PEMF showed significant upregulations of collagen I, alkaline phosphatase, and osteocalcin	2018	Poh et al. [18]
5	H4 glioma cells	Frequency of 7 Hz Intensity of 30 mT	Cell apoptosis	LFPEMF stimulation of H4 glioma cell cultures induced apoptosis in exposed cells.	2018	Kaszuba-Zwoińska et al. [38]
6	Mesenchymal stem cells (hMSCs)	Frequency of 75 Hz, the intensity peak of 1.5 mT	Gene expression	The exposure to PEMFs did not produce any change on notch-related genes	2017	Bagheri et al. [20]
7	Human umbilical vein endothelial cells (HUVECs)	The frequency of 50 Hz Intensity of 2.25 mT	Cell proliferation Gene expression Protein expression	Proteins and mRNA expression levels of Akt, mTOR, and TGF-*β*1 were elevated	2017	Cheng et al. [59]
8	Human mesenchymal stem cells (MSCs)	Frequency of 15 Hz Flux densities between 1–4 mT.	Gene expression	Brief and single exposures to low amplitude PEMFs were most effective at stimulating MSC chondrogenesis.	2017	Parate et al. [21]

The article "Evaluation of Pulsed Electromagnetic Field Effects: A Systematic Review and Meta-Analysis on Highlights of Two Decades of Research In Vitro Studies" was published in 2021. Journal: Biomed Res Int.

**Table 3:** Human cell studies: PEMF exposure conditions used in in vitro studies.

No.	Cell line	Frequencies and intensities	Cell response analysis	Result	Year	First author
9	MCF-7	Frequencies of 2122.24, 1970.56, 2072.32, and 2648.64 Hz	Cell viability	There was a significant effect on MCF-7 cells after treatment with PEMF at the resonant frequencies of the genes of RICTOR, PPARG, and NBN CHEK2	2017	Alcantara et al. [43]
10	U937 cells (leukemia cell line)	Frequency of 50 Hz Intensity of 45 mT	Cell viability protein expression	There were no significant differences in the expression level of calmodulin between control- and only MF-treated samples	2017	Wojcik-Piotrowicz et al. [46]
11	Human bone marrow stromal cells (hBMSCs)	Pulse frequency of 3.8 kHz	Enzyme activity Signal transduction Pathway Gene expression	PEMF regulated preosteoblast gene expression, and notably, the transforming growth factor-beta (TGF-*β*) signaling pathway and microRNA 21 (miR21) were the most highly regulated	2017	Selvamurugan et al. [25]
25	Peripheral blood mononuclear cells (PBMCs)	Frequency of 75 Hz Intensity of 3 mT	Gene expression	LF-PEMF modulated gene expression.	2017	Capelli et al. [57]
12	Human bone marrow mesenchymal stem cells (hBM-MSCs)	Frequency of 60 Hz Intensity of 10 mT	Protein expression	After exposure to only PEMF, the expression of proteins slightly increased, but there was no significant difference when compared to the nonexposed groups.	2016	Choi et al. [26]
13	Human glioblastoma U87 cell line	Frequencies of 50 Hz and 100 Hz intensities of 10 mT and 5 mT	Cell viability Cell morphology Protein expression	A significant increase in the number of cells after 24 h exposure to 50 Hz, 100 G. A dramatic decrease in cells exposed to 100 Hz, 100 G, and 10 Hz, 50 G EMFs compared with controls	2016	Akbarnejad et al. [3]
14	Human glioblastoma cell line (T98G).	Frequency of 75 Hz Intensity of 2 mT	Cell proliferation, cell apoptosis	miR-421 expression significantly increased over the control after PEMF alone.	2016	Pasi et al. [39]

**Table 4:** Human cell studies: PEMF exposure conditions used in in vitro studies.

No.	Cell line	Frequencies and intensities	Cell response analysis	Result	Year	First author
15	Periodontal ligament stem cells (PDLSCs)	Pulsed burst frequency of 15 Hz Intensities of 0.6, 1.2, 1.8, 2.4, and 3.0 mT	Cell proliferation Cell differentiation Gene expression Protein expression	No influence on cell proliferation. PEMF appeared to stimulate the earlier onset of osteogenic differentiation of PDLSCs and upregulated the gene expression of Runx2, ALP, and OPN compared with the sham group.	2016	Wang et al. [32]
16	Human mesenchymal stem cells (MSCs)	Frequency of 50 Hz Intensity of 0.6 mT	Cell viability Cell differentiation Gene expression	PEMFs upregulated genes related to Ca^2+^ signaling, proliferation, and neurogenic differentiation	2016	Lim et al. [11]
17	Human tendon stem cells (hTSCs)	Frequency of 10–30 Hz Intensity of 0.5–1.5 mT	Cell morphology Cell viability Cell proliferation Cell apoptosis Gene expression	PEMF did not cause any significant changes in proliferation, viability, and morphology.	2016	Randelli et al. [33]
18	Human dental pulp stem cells (hDPSCs) Schwann-like cells	Frequency of 50 Hz Intensity of 1 mT	Gene expression	Group treated to PEMF showed significantly greater P75NTR mRNA expression than the control group	2016	Hei et al. [34]
19	HeLa, HEK293, MCF7, and AGS	Frequency of 75 Hz Intensities of 2, 4, and 6 mT	Cell proliferation	Cell proliferations of all four different cell lines also showed an increase in PEMF exposure until 4 mT, but not at 6 mT.	2016	Cho et al. [44]
20	Human annulus fibrosus (AF) cells Nucleus pulposus (NP) cells	Frequency of 3,850 Hz Intensity of 1.19 mT	Gene expression	PEMF alone had no effect on gene expression.	2016	Miller et al. [62]

The article "Evaluation of Pulsed Electromagnetic Field Effects: A Systematic Review and Meta-Analysis on Highlights of Two Decades of Research In Vitro Studies" was published in 2021. Journal: Biomed Res Int.

**Table 5:** Human cell studies: PEMF exposure conditions used in in vitro studies.

No.	Cell line	Frequencies and intensities	Cell response analysis	Result	Year	First author
21	Human dermal fibroblasts (HDF), human epidermal keratinocytes (HEK), and human mononuclear cells (HMNC)	Pulse frequency of 1 kHz, intensity of 6.7 A/m	Gene expression	PEMF treatment changed the relative amount of messenger (m) RNA encoding enzymes involved in heme catabolism and removal of reactive oxygen species.	2015	Kubat et al. [60]
22	Acute lymphoblastic leukemia (CEM/C2), B-cell lymphoma (SU-DHL-4), colorectal adenocarcinoma (COLO-320DM), breast adenocarcinoma (MDABM-468), and ductal carcinoma (ZR-75-1)	Frequencies of 15 Hz, 125 Hz, and 625 Hz intensity of 5 mT	Cell morphology, cell viability, and cell apoptosis	A PEMF of 125 Hz and 625 Hz for 24 h–48 h increased proliferation activity in the 2 types of cancer cell lines used	2015	Loja et al. [48]
23	Human neuroblastoma SH-SY5Y cells	Frequency of 75 Hz Intensity of 2 mT	Enzymatic activity, cell proliferation, cell viability, and cell apoptosis	Basal MnSOD specific activity was higher in PEMF stimulated cells when compared to cells not treated with PEMF	2015	Osera et al. [42]
24	Human bone marrow stromal cells (hBMSCs)	Frequency of 200 Hz Intensities of 0.6, 1 tesla	Cell proliferation Cell differentiation	Proliferation and the osteogenic differentiation of hBMSCs were increased	2014	Fu et al. [31]
25	Human amniotic epithelial cells (AECs)	Frequency of 50 Hz Intensity of 1 mT	Cell differentiation Gene expression Protein expression	The PEMF stimulation could induce osteogenic differentiation, as shown by the expression of osteoblast-specific genes and proteins including alkaline phosphatase and osteocalcin	2014	Wang et al. [35]

**Table 6:** Human cell studies: PEMF exposure conditions used in in vitro studies.

No.	Cell line	Frequencies and intensities	Cell response analysis	Result	Year	First author
26	Human tendon cells (hTCs)	Intensities of 1.5 and 3 mT	Cell viability Cell proliferation Gene expression	Proliferation and the viability of hTCs were enhanced by PEMF	2014	de Girolamo et al. [61]
27	Human umbilical cord-derived Mesenchymal stem cells	Frequency of 75 Hz, intensity of 1.8-3 mT	Cell morphology Gene expression	Morphological data showed that the treatment with PMEF reduced the time to obtain cell differentiation.	2013	Esposito et al. [36]
28	Human disc cells	Frequency of 15 Hz. Intensity of 1.6 mT	Gene expression Protein expression	BMP-7 and BMP-2 were upregulated by PEMF	2013	Okada et al. [63]
29	Tendon cells (TCs) (human)	Frequency of 75 Hz, intensity of 1.5 mT	Cell morphology, cell viability, cell apoptosis, and gene expression	PEMF exposure is not cytotoxic and is able to stimulate TCs' proliferation	2013	de Girolamo et al. [15]
30	Human disc cells (intervertebral disc (IVD))	Frequency of 15 Hz Intensity of 1.6 mT	Gene expression Protein expression	mRNA expression of BMP-2 was upregulated by PEMF alone	2013	Okada et al. [64]
31	MCF7, MCF10	Frequencies of 20 and 50 Hz Intensities of 2.0, 3.0, and 5.0 mT	Cell apoptosis	MCF7 cancer cells were particularly vulnerable to 3 mT PEMFs.	2013	Crocetti et al. [45]
32	Bone marrow MSCs (BM-MSCs) Adipose tissue mesenchymal stem cells (ASC)	Frequency of 75 Hz, intensity of 2 mT	Cell viability Cell proliferation Cell morphology Cell apoptosis Gene expression Cell differentiation	After PEMF exposure, in comparison with ASCs, BM-MSCs showed an increase in cell proliferation	2013	Ceccarelli et al. [19]
33	Human osteogenic sarcoma SaOS-2 Bone marrow-derived human MSCs	Frequency of 15 Hz, intensity of 0.1 mT	Cell proliferation Gene expression	PEMF caused a minor increase in expression of osteogenic markers of MSCs	2012	Kaivosoja et al. [50]

The article "Evaluation of Pulsed Electromagnetic Field Effects: A Systematic Review and Meta-Analysis on Highlights of Two Decades of Research In Vitro Studies" was published in 2021. Journal: Biomed Res Int.

**Table 7:** Human cell studies: PEMF exposure conditions used in in vitro studies.

No.	Cell line	Frequencies and intensities	Cell response analysis	Result	Year	First author
34	Human mesenchymal stem cell osteoblast	Frequencies of 5, 25, 50, 75, 100, and 150 Hz, intensity of 1.1 mT,	Cell differentiation	Levels of human mesenchymal stem cell differentiation changed by PEMF	2012	Luo et al. [37]
35	Stromal cells of human bone marrow (BMSC)	Frequency of 75 Hz, intensity of 1.8-3 mT	Gene expression, cell differentiation	The cells treated with PEMF began differentiation earlier than untreated cells.	2012	Esposito et al. [24]
36	Human breast carcinoma cells (T47D)	Frequencies of 100, 217 Hz intensity of 0.1 mT	Cell proliferation, cell viability, cell morphology, protein expression, and ROS production	PEMF induced a time-dependent decrease in cell growth after 72 h	2012	Sadeghipour et al. [49]
37	Human peripheral blood mononuclear cell (PBMC)	Frequency of 7 Hz flux density of 30 mT	Cell apoptosis	PEMF induced apoptosis in PBMC	2011	Kaszuba-Zwoińska et al. [58]
38	Bone marrow mesenchymal stem cells (BMMSCs)	Frequency of 15 Hz flux density of 1.8 mT	Cell proliferation Cell apoptosis Gene expression Protein expression	PEMF treated cells also showed greater MMP-2 expression compared to unstimulated cells.	2011	Griffin et al. [27]
39	Human bone marrow-derived stromal cell (BMSC) Human fetal preosteoblasts (SVHFO)	Frequency of 15 Hz Flux density of 0.1 mT	Cell proliferation Cell differentiation Gene expression Signal pathway	PEMF treatment increased mRNA levels of bone morphogenetic protein 2, transforming growth factor-beta 1, osteoprotegerin, matrix metalloproteinase-1 and -3, osteocalcin, and bone sialoprotein	2010	Jansen et al. [28]
40	Osteoblast-like cell cultures (MG-63)	Frequency of 75 Hz Flux density of 3 mT	Gene expression	PEMFs induced the upregulation of important genes related to bone formation genes, however, PEMF induced downregulation of genes related to the degradation of extracellular matrix		Sollazzo et al. [53]

The article "Evaluation of Pulsed Electromagnetic Field Effects: A Systematic Review and Meta-Analysis on Highlights of Two Decades of Research In Vitro Studies" was published in 2021. Journal: Biomed Res Int.

**Table 8:** Human cell studies: PEMF exposure conditions used in in vitro studies.

No.	Cell line	Frequencies and intensities	Cell response analysis	Result	Year	First author
41	Human osteoblast-like Saos-2 cells	Frequency of 15 Hz flux density of 2 mT	Gene expression Protein expression	PEMF induced increase in RANKL mRNA expression	2010	Borsje et al. [51]
42	Bone marrow mesenchymal stem cells (BMMSCs)	Frequency of 15 Hz flux density of 1.8 mT	Cell proliferation Gene expression	Exposure of BMMSCs to PEMFs increased cell proliferation	2010	Sun et al. [29]
43	Human mesenchymal stem cells (hMSCs)	Frequency of 7.5 Hz flux density of 0.13 mT	Cell proliferation Cell differentiation Gene expression	The expressions of osteogenic genes, including Runx2/Cbfa1 and ALP, were modulated by PEMF exposure.	2009	Tsai et al. [22]
44	Human bone marrow mesenchymal stem cells (BMMSC)	Frequency of 15 Hz flux density of 1.8 mT	Cell morphology Cell proliferation Cell differentiation	PEMF exposure could enhance the BMMSC cell proliferation	2009	Sun et al. [30]
45	SaOS-2 osteoblast-like cells	Frequency of 15 Hz	Cell viability Cell proliferation Cell differentiation	PEMF stimulation did not affect cell number, however, increased ALP activity	2008	Martino et al. [7]
46	Human chondrocyte	Frequency of 21.2 MHz	Cell viability	PEMF exposure increase cell viability	2007	Štolfa et al. [66]
47	Primary human mesenchymal stem cells (MSCs), human chondrocyte	Frequency of 30 Hz, intensity of 35 *μ*T	Gene expression	PEMF altered the gene expression of a limited number of gene products in human mesenchymal stem cells and human chondrocytes.	2007	Walther et al. [23]
48	Human promyelocytic leukemia HL-60 cells	Frequency of 0.25 Hz 0.25–4.5 T peak magnetic field strength	Cell viability signal transduction	PEMF did not alter the cell viability or content of cAMP	2006	Sontag and Kalka [47]
49	A human osteosarcoma (cell line) SaOS-2	Frequency of 15 Hz Intensity of 1.6 mT	Cell Proliferation Cell differentiation	PEMF reduced proliferation and increased differentiation in SaOS-2 cell line	2005	Hannay et al. [52]
50	MG-63 human osteosarcoma cells	Frequency of 75 Hz, intensity of 2.3 mT	Cell proliferation Gene expression	The PEMF increased [3H]-thymidine incorporation	2005	Mattei et al. [54]

The article "Evaluation of Pulsed Electromagnetic Field Effects: A Systematic Review and Meta-Analysis on Highlights of Two Decades of Research In Vitro Studies" was published in 2021. Journal: Biomed Res Int.

**Table 9:** Human cell studies: PEMF exposure conditions used in in vitro studies.

No.	Cell line	Frequencies and intensities	Cell response analysis	Result	Year	First author
51	Human astrocytoma cell line U-373 MG	Frequency of 50 Hz, intensity of 3 mT	Cell proliferation	PEMF did not cause cell proliferation or cell death	2001	Pessina et al. [40]
52	Sympathetic neuronal-like PC6 cells	Frequency of 2 Hz, intensity of 0.3 mT	Cell proliferation, cell differentiation	Proliferation was unaffected by PEMF	2001	Shah et al. [67]
53	Human atrophic nonunion cell culture Hypertrophic nonunion cell culture	Frequency of 15 Hz, intensity of 1.8 mT	Cell morphology Cell proliferation Cell differentiation	PEMF resulted in a change in morphologic features of cells.	2001	Guerkov et al. [65]
54	Human astrocytoma cell line U-373 MG cells	Frequency of 50 Hz, intensity of 3 mT	Cell proliferation Ca^2+^ concentration	After the cells were exposed to EMFs, the basal [Ca^2+^]i levels increased	2000	Aldinucci et al. [41]
55	TE-85 human osteosarcoma cells MG-63 human osteosarcoma cells Human normal osteoblast cells (NHOC)	Frequency of 15 Hz, intensity of 1.8 mT	Cell proliferation	The cells increase their proliferation when exposed to PEMF	1999	De Mattei et al. [55]
56	MG63 human osteoblast-like cells	Frequency of 75 Hz, intensity of 2.3 mT	Cell proliferation, cell differentiation	PEMF caused a reduction in cell proliferation and an increase ALP activity	1999	Lohmann et al. [4]

**Table 10:** Rat/mouse cells: cellular response (presence or absence) for cultured rat/mouse cells.

No.	Cell line	Frequency and intensity	Cell response analysis	Result	Year	Authors
57	MC3T3-E1	Flux density of either 0.1 or 0.4 mT. Frequency of 10 Hz.	Signal transduction pathway, cell proliferation, cell differentiation	The activation of mTOR, increased, BrdU uptake was increased, and ALPase activity was not observed.	2019	Miyamoto et al. [91]
58	RAW264.7	Frequency of 75 Hz, flux density of 1 mT.	Cell viability, cell differentiation, gene expression, protein expression	The results revealed no significant difference between groups stimulated by PEMF alone and control group.	2019	Pi et al. [78]
59	Oligodendrocyte precursor cells (OPCs)	Frequency of 50 Hz, intensity of 1.8 mT.	Cell differentiation, protein expression, gene expression	PEMF promoted the differentiation of OPCs. PEMF upregulated the expression level of miR-219-5p and downregulated the expression level of Lingo1 during the differentiation of OPCs.	2019	Yao et al. [5]
60	Tendon stem and progenitor cells (TDSPCs)	Frequency of 125 kHz, intensity of 82 mT	Cell viability, cell apoptosis	The exposure to PEMF alone did not effect on the viability and apoptosis of cells	2019	Gehwolf et al. [70]
61	MC3T3-E1 subclone 4 cells	Frequency of 50 Hz, intensity of 0.60 mT	Cell morphology, cell viability, cell proliferation, Ca^2+^ concentration, gene expression	PEMF influenced cell proliferation, did not significantly influence cellular viability, and affected osteogenic differentiation on mRNA level	2019	Suryani et al. [92]
62	Bone marrow-derived mesenchymal stem cells (BMSCs) (rat)	50 Hz, 1 mT	Cell proliferation, gene expression	S100, GFAP, and NGF mRNA expression levels were higher on days 5, 7, and 10 of culture.		Seo et al. [73]
63	C3H10T1/2 mesenchymal cells	Frequency of 30 Hz, intensities of 0.1, 1, 2, or 10 mT	Cell proliferation, cell differentiation, Ca^2+^ concentration, gene expression, protein expression	Cell proliferation was promoted, and intracellular Ca^2+^ during the process of cell differentiation was increased. The expression of ALP, OSX, Wnt1, phospho-Lrp6, and b-catenin was increased	2018	Wu et al. [71]

The article "Evaluation of Pulsed Electromagnetic Field Effects: A Systematic Review and Meta-Analysis on Highlights of Two Decades of Research In Vitro Studies" was published in 2021. Journal: Biomed Res Int.

**Table 11:** Rat/mouse cells: cellular response (presence or absence) for cultured rat/mouse cells.

No.	Cell line	Frequency and intensity	Cell response analysis	Result	Year	Authors
64	RAW264.7 cells	Frequency of 15 Hz intensities of 0.5, 1, 2, and 3 mT	Cell apoptosis, gene expression	Gene expression of RANK, NFATc1, TRAP, CTSK, BAX, and BAX/BCL was significantly decreased by 0.5 mT PEMF, but increased by 3 mT	2017	Wang et al. [79]
65	Spermatogonia germ cell line, (GC-1), spermatocyte cell line (GC-2)	Frequencies of 2, 50, and 120 Hz, intensity of 2.5 mT	Cell proliferation, cell morphology, cellular oxidative stress, protein expression, cell viability	PEMF resulted in elongated and fibroblast-like shapes in GC-1 spg cells. PEMF increased the total p53 protein level in GC-2 spd cells.	2017	Solek et al. [83]
66	Adipose-derived stem cells (ADSCs) isolated	Frequency of 7 Hz, flux density of 30 mT	Cell apoptosis	Exposure to PEMF resulted in a significant increase in the proportion of apoptotic cells	2017	Baranowska et al. [69]
67	Primary rat nucleus pulposus cells	Frequency of 2 Hz, intensities of 0.5, 1.0, 2.0, and 3.0 A/m	Cell morphology, cell viability, protein expression	Stimulation of nucleus pulposus cells with LF-PEMFs did not appear to affect cell morphology or nucleus pulposus cell IL-1*β* and TNF-*α* expression levels.	2017	Zou et al. [84]
68	Mouse osteosarcoma cell line (LM8 cells)	Frequency of 200 Hz, flux density of 5 mT	Ca^2+^ concentration, cell apoptosis	The level of intracellular Ca^2+^ after PEMF treatment was significantly higher.	2017	Muramatsu et al. [85]
69	C2C12 myoblasts	Frequency of 100 Hz, flux density of 1 mT	Cell proliferation, cell apoptosis, signal transduction, pathway, protein expression	Increase of proliferation, no influence on the apoptosis the phosphorylation level of extracellular, signal-regulated kinase (ERK) was significantly increased, while p38 MAPK and c-Jun N-terminal kinase (JNK) pathways were not affected.	2016	Xu et al. [96]
70	Bone marrow stem cells (BMSCs)	Frequency of 20 Hz, flux density of 2 mT	Gene expression, cell differentiation	PEMFs significantly promoted the activity of ALP in the BMSCs and mRNA expression of osteogenic proteins	2015	Lu et al. [74]

The article "Evaluation of Pulsed Electromagnetic Field Effects: A Systematic Review and Meta-Analysis on Highlights of Two Decades of Research In Vitro Studies" was published in 2021. Journal: Biomed Res Int.

**Table 12:** Rat/mouse cells: cellular response (presence or absence) for cultured rat/mouse cells.

No.	Cell line	Frequency and intensity	Cell response analysis	Result	Year	Authors
71	Rat bone marrow-derived stem cells	Frequency of 75 Hz Intensities of 1, 2, or 5 mT	Cell proliferation	PEMF stimulation did not cause significant changes in rat BMSC proliferation	2015	Wang et al. [75]
72	The murine MN9D dopaminergic cell line	Frequency of 5 Hz	Cell morphology	PEMF signals increased cell body width	2014	Lekhraj et al. [68]
73	Primary culture osteoblastic cells	Intensities of 0.06 and 0.2 mT	Cell proliferation Cell viability Cell differentiation Cell morphology	Control group had a higher cell proliferation than 0.06 and 0.2 mT PEMF groups	2013	Emes et al. [86]
74	RAW 264.7 macrophage-like cells (murine)	Frequencies of 5.1 Hz, 7.8 Hz, 10.8 Hz, 15.6 Hz, 20.8 Hz, 23.4 Hz, or 30 Hz. Intensity of 4 mT	Signaling pathways Gene expression	Cells exposed to PEMF demonstrated changes in the downregulation of NFkB	2013	Ross and Harrison [80]
75	PC12 and NR8383 rat alveolar macrophages	Frequency of 0.172 Hz Intensity of 700 mT	Signal pathway Enzyme activity	PEMF induced activation of ERK1/2 in PC12 cells	2013	Tada-Aki et al. [81]
76	Rat brain cortical neurons, PC12, U87MG cells	Frequency of 75 Hz, intensity of 1.5 mT	Gene expression Cell apoptosis	PEMF treatment induced an upregulation of A3ARs, A_2_ARs	2012	Vincenzi et al. [82]
77	C3H10T1/2 cells Immortalized calvarial cells iCALs	Frequency of 1000 Hz	Cell differentiation Cell proliferation Gene expression Protein expression	PEMF stimulation augmented osteopontin and osteocalcin expression	2012	Teven et al. [72]
78	Mesenchymal stem cells (MSCs)	Frequency of 50 Hz, intensity of 10 mT	Cell viability, cell proliferation	PEMF increases the proliferation of MSC cells.	2012	Li et al. [76]

The article "Evaluation of Pulsed Electromagnetic Field Effects: A Systematic Review and Meta-Analysis on Highlights of Two Decades of Research In Vitro Studies" was published in 2021. Journal: Biomed Res Int.

**Table 13:** Rat/mouse cells: cellular response (presence or absence) for cultured rat/mouse cells.

No.	Cell line	Frequency and intensity	Cell response analysis	Result	Year	Authors
79	The murine osteoblast-like cell line MC3T3-E1	Frequency of 0.5 Hz, intensities of 0.17 mT and 1.33 mT	Cell proliferation Cell differentiation Gene expression Protein expression	The proliferation and differentiation of cells in PEMF exposure groups changed, COL-I and Cbfa1 mRNA expression and BMP2/4 and Smad1/5/8 protein expression did not change.	2011	Li et al. [93]
80	Rat basophilic leukemia cells (RBL-2H3)	Frequency of 8 kHz, intensity of 200 mT	Cell morphology Cell proliferation Gene expression	PEMF Stimulation led to increased cell proliferation	2010	Choi et al. [97]
81	Rat bone marrow cells	Frequency of 8 Hz, intensity of 3.8 mT	Gene expression	No statistically significant difference was found between the PEMF group and the control group	2010	Chen et al. [98]
82	Neural stem cells (NSCs)	Frequency of 0.1 Hz, intensities of 0.5, 1.0, 3.0, 4.0, 5.0, 6.0, 8.0, and 10.0 T	Cell proliferation Cell differentiation	Exposure of NSCs to PEMFs changed cell proliferation	2009	Meng et al. [77]
83	Osteoblast-like MC3T3-E1 cells Primary osteoblast cells	Frequency of 48 Hz Intensity of 1.55 mT	Cell proliferation Cell differentiation	PEMF treatment accelerated the cell proliferation and promoted cell differentiation of the primary osteoblast cell.	2008	Wei et al. [87]
84	Rat primary osteoblastic cells	Frequency of 3.8 kHz	Cell proliferation Gene expression	Continuous daily 4 h treatment with PEMF alone increased expression of osteoblast marker genes	2007	Selvamurugan et al. [88]
85	A rat osteogenic cell line	Physio-stim® PEMF signals	Signal pathway	PEMF induced rapid phosphorylation reactions of Intracellular signaling molecules	2006	Schnoke and Midura [89]
86	Murine Preosteoblasts MC3T3-E1 Fibroblast cell lines	Frequency of 3850 Hz Intensity of 0.4 mT	Signal transduction pathway	mTOR pathway was activated within minutes of PEMF exposure	2006	Patterson et al. [95]

**Table 14:** Rat/mouse cells: cellular response analysis for cultured rat/mouse cells.

No.	Cell line	Frequency and intensity	Cell response analysis	Result	Year	Authors
87	Pheochromocytoma cells (PC12)	Frequency of 0.25 Hz Intensity of 0.25–4.5 T	Cell viability Signal transduction	PEMF did not alter the cell viability or content of cAMP	2006	Sontag and Kalka [47]
88	Osteoblast-like cells	Frequency of 15 Hz, intensity of 0.1 mT	Cell proliferation Cell differentiation Gene expression	PEMF of osteoblasts accelerated cellular proliferation, but did not affect the cellular differentiation	2004	Chang et al. [90]
89	MLO-Y4 osteocyte-like cells ROS 17/2.8 cells	Frequency of 15 Hz, intensity of 1.6 mT	Cell proliferation, cell differentiation Protein expression Enzyme activity	PEMF did not affect cell number, osteocalcin mRNA, or osteocalcin protein	2003	Lohmann et al. [101]
90	Osteoblast-like MC3T3-E1 cell line	Frequency of 15 Hz, intensity of 7 mT	Cell proliferation Cell differentiation	PEMF treatment accelerated cellular proliferation and enhanced cellular differentiation.	2002	Diniz et al. [94]

The article "Evaluation of Pulsed Electromagnetic Field Effects: A Systematic Review and Meta-Analysis on Highlights of Two Decades of Research In Vitro Studies" was published in 2021. Journal: Biomed Res Int.

**Table 15:** Other species cell studies.

No.	Cell line	Frequency and intensity	Cell response analysis	Result	Year	Authors
91	Intervertebral discs (IVDs) from bovine caudal spines	Pulse frequency of 3850 Hz	Protein expression, signal pathway	Overall p65 expression was increased, and P38 expression was not influenced.	2019	Tang et al. [99]
92	Rabbit adipose-derived mesenchymal stem cells (AD-MSCs)	Frequencies of 25 Hz and 50 Hz, intensity of 1.6 mT	Cell proliferation Gene expression	PEMF did not cause any significant increase in SOX9 mRNA productions	2016	Kavand et al. [100]

## Data Availability

Access to data is restricted due to ethical concerns.

## References

[1] Maziarz A., Kocan B., Bester M. (2016). How electromagnetic fields can influence adult stem cells: positive and negative impacts. *Stem Cell Research & Therapy*.

[2] Markov M., Klauenberg B. J., Miklavcic D. (2000). Dosimetry of magnetic fields in the radiofrequency range. *Radio Frequency Radiation Dosimetry*.

[3] Akbarnejad Z., Eskandary H., Vergallo C. (2017). Effects of extremely low-frequency pulsed electromagnetic fields (ELF-PEMFs) on glioblastoma cells (U87). *Electromagnetic biology and medicine.*.

[4] Lohmann C., Schwartz Z., Liu Y. (2000). Pulsed electromagnetic field stimulation of MG63 osteoblast-like cells affects differentiation and local factor production. *Journal of Orthopaedic Research.*.

[5] Yao F., Li Z., Cheng L., Zhang L., Zha X., Jing J. (2019). Low frequency pulsed electromagnetic field promotes differentiation of oligodendrocyte precursor cells through upregulation of miR-219-5p in vitro. *Life sciences.*.

[6] Ganesan K., Gengadharan A. C., Balachandran C., Manohar B. M., Puvanakrishnan R. (2009). Low frequency pulsed electromagnetic field—a viable alternative therapy for arthritis. *Indian Journal of Experimental Biology*.

[7] Martino C. F., Belchenko D., Ferguson V., Nielsen-Preiss S., Qi H. J. (2008). The effects of pulsed electromagnetic fields on the cellular activity of SaOS-2 cells. *Bioelectromagnetics*.

[8] Delle Monache S., Angelucci A., Sanità P. (2013). Inhibition of angiogenesis mediated by extremely low-frequency magnetic fields (ELF-MFs). *PLoS One.*.

The article "Evaluation of Pulsed Electromagnetic Field Effects: A Systematic Review and Meta-Analysis on Highlights of Two Decades of Research In Vitro Studies" was published in 2021. Journal: Biomed Res Int.

[9] Furuya-Kanamori L., Xu C., Lin L. (2020). _P_ value -driven methods were underpowered to detect publication bias: analysis of Cochrane review meta-analyses. *Journal of clinical epidemiology.*.

[10] Ross C. L., Ang D. C., Almeida-Porada G. (2019). Targeting mesenchymal stromal cells/pericytes (MSCs) with pulsed electromagnetic field (PEMF) has the potential to treat rheumatoid arthritis. *Frontiers in immunology.*.

[11] Lim K. T., Seonwoo H., Choi K. S. (2016). Pulsed-electromagnetic-field-assisted reduced graphene oxide substrates for multidifferentiation of human mesenchymal stem cells. *Advanced Healthcare Materials.*.

[12] Semenov I., Xiao S., Pakhomov A. G. (2013). Primary pathways of intracellular Ca^2 +^ mobilization by nanosecond pulsed electric field. *Biochimica et Biophysica Acta (BBA)-Biomembranes*.

[13] Hinrikus H., Karpowicz J., Naarala J. (2018). *Electromagnetic Fields in Biology and Medicine*.

[14] Vadalà M., Morales-Medina J. C., Vallelunga A., Palmieri B., Laurino C., Iannitti T. (2016). Mechanisms and therapeutic effectiveness of pulsed electromagnetic field therapy in oncology. *Cancer medicine.*.

[15] De Girolamo L., Stanco D., Galliera E. (2013). Low frequency pulsed electromagnetic field affects proliferation, tissue-specific gene expression, and cytokines release of human tendon cells. *Cell biochemistry and biophysics.*.

[16] Daish C., Blanchard R., Duchi S. Design, fabrication and validation of a precursor pulsed electromagnetic field device for bone fracture repair.

[17] Yin Y., Chen P., Yu Q., Peng Y., Zhu Z., Tian J. (2018). The effects of a pulsed electromagnetic field on the proliferation and osteogenic differentiation of human adipose-derived stem cells. *Medical science monitor: international medical journal of experimental and clinical research*.

[18] Poh P. S., Seeliger C., Unger M., Falldorf K., Balmayor E. R., van Griensven M. (2018). Osteogenic effect and cell signaling activation of extremely low-frequency pulsed electromagnetic fields in adipose-derived mesenchymal stromal cells. *Stem cells international.*.

[19] Ceccarelli G., Bloise N., Mantelli M. (2013). A comparative analysis of the in vitro effects of pulsed electromagnetic field treatment on osteogenic differentiation of two different mesenchymal cell lineages. *Bio Research open access.*.

[20] Bagheri L., Pellati A., Rizzo P. (2018). Notch pathway is active during osteogenic differentiation of human bone marrow mesenchymal stem cells induced by pulsed electromagnetic fields. *Journal of tissue engineering and regenerative medicine.*.

[21] Parate D., Franco-Obregón A., Fröhlich J. (2017). Enhancement of mesenchymal stem cell chondrogenesis with short-term low intensity pulsed electromagnetic fields. *Scientific reports*.

The article "Evaluation of Pulsed Electromagnetic Field Effects: A Systematic Review and Meta-Analysis on Highlights of Two Decades of Research In Vitro Studies" was published in 2021. Journal: Biomed Res Int.

[22] Tsai M. T., Li W. J., Tuan R. S., Chang W. H. (2009). Modulation of osteogenesis in human mesenchymal stem cells by specific pulsed electromagnetic field stimulation. *Journal of orthopaedic research*.

[23] Walther M., Mayer F., Kafka W., Schütze N. (2007). Effects of weak, low-frequency pulsed electromagnetic fields (BEMER type) on gene expression of human mesenchymal stem cells and chondrocytes: an in vitro study. *Electromagnetic biology and medicine.*.

[24] Esposito M., Lucariello A., Riccio I., Riccio V., Esposito V., Riccardi G. (2012). Differentiation of human osteoprogenitor cells increases after treatment with pulsed electromagnetic fields. *In vivo*.

[25] Selvamurugan N., He Z., Rifkin D., Dabovic B., Partridge N. C. (2017). Pulsed electromagnetic field regulates micro RNA 21 expression to activate TGF-*β* signaling in human bone marrow stromal cells to enhance osteoblast differentiation. *Stem cells international*.

[26] Choi Y. K., Urnukhsaikhan E., Yoon H. H. (2017). Combined effect of pulsed electromagnetic field and sound wave on in vitro and in vivo neural differentiation of human mesenchymal stem cells. *Biotechnology progress.*.

[27] Griffin M., Iqbal S. A., Sebastian A., Colthurst J., Bayat A. (2011). Degenerate wave and capacitive coupling increase human MSC invasion and proliferation while reducing cytotoxicity in an in vitro wound healing model. *PLoS One.*.

[28] Jansen J. H., van der Jagt O. P., Punt B. J. (2010). Stimulation of osteogenic differentiation in human osteoprogenitor cells by pulsed electromagnetic fields: an in vitro study. *BMC musculoskeletal disorders.*.

[29] Sun L. Y., Hsieh D. K., Lin P. C., Chiu H. T., Chiou T. W. (2010). Pulsed electromagnetic fields accelerate proliferation and osteogenic gene expression in human bone marrow mesenchymal stem cells during osteogenic differentiation. *Bioelectromagnetics: Journal of the Bioelectromagnetics Society, The Society for Physical Regulation in Biology and Medicine, The European Bioelectromagnetics Association.*.

[30] Sun L. Y., Hsieh D. K., Yu T. C. (2009). Effect of pulsed electromagnetic field on the proliferation and differentiation potential of human bone marrow mesenchymal stem cells. *Bioelectromagnetics*.

[31] Fu Y.-C., Lin C.-C., Chang J.-K. (2014). A novel single pulsed electromagnetic field stimulates osteogenesis of bone marrow mesenchymal stem cells and bone repair. *PLoS One.*.

[32] Wang T., Wang P., Cao Z. (2017). Effects of BMP9 and pulsed electromagnetic fields on the proliferation and osteogenic differentiation of human periodontal ligament stem cells. *Bioelectromagnetics.*.

The article "Evaluation of Pulsed Electromagnetic Field Effects: A Systematic Review and Meta-Analysis on Highlights of Two Decades of Research In Vitro Studies" was published in 2021. Journal: Biomed Res Int.

[33] Randelli P., Menon A., Ragone V. (2016). Effects of the pulsed electromagnetic field PST® on human tendon stem cells: a controlled laboratory study. *BMC Complementary and Alternative Medicine.*.

[34] Hei W. H., Kim S., Park J. C. (2016). Schwann-like cells differentiated from human dental pulp stem cells combined with a pulsed electromagnetic field can improve peripheral nerve regeneration. *Bioelectromagnetics.*.

[35] Wang Q., Wu W., Han X. (2014). Osteogenic differentiation of amniotic epithelial cells: synergism of pulsed electromagnetic field and biochemical stimuli. *BMC musculoskeletal disorders.*.

[36] Esposito M., Lucariello A., Costanzo C. (2013). Differentiation of human umbilical cord-derived mesenchymal stem cells, WJ-MSCs, into chondrogenic cells in the presence of pulsed electromagnetic fields. *in vivo*.

[37] Luo F., Hou T., Zhang Z., Xie Z., Wu X., Xu J. (2012). Effects of pulsed electromagnetic field frequencies on the osteogenic differentiation of human mesenchymal stem cells. *Orthopedics.*.

[38] Kaszuba-Zwoińska J., Nowak B., Guzdek P., Gil K. Cell viability changes in cultured H4 glioma cells upon low frequency pulsed electromagnetic field (7Hz, 30mT) exposure in flow cytometry analysis.

[39] Pasi F., Fassina L., Mognaschi M. E. (2016). Pulsed electromagnetic field with temozolomide can elicit an epigenetic pro-apoptotic effect on glioblastoma T98G cells. *Anticancer research.*.

[40] Pessina G., Aldinucci C., Palmi M. (2001). Pulsed electromagnetic fields affect the intracellular calcium concentrations in human astrocytoma cells. *Bio electro magnetics*.

[41] Aldinucci C., Palmi M., Sgaragli G. (2000). The effect of pulsed electromagnetic fields on the physiologic behaviour of a human astrocytoma cell line. *Biochimica et Biophysica Acta (BBA)-Molecular Cell Research*.

[42] Osera C., Amadio M., Falone S. (2015). Pre-exposure of neuroblastoma cell line to pulsed electromagnetic field prevents H2O2-induced ROS production by increasing MnSOD activity. *Bioelectromagnetics.*.

[43] Alcantara D. Z., Soliman I. J. S., Pobre R. F., Naguib R. N. (2017). Effects of pulsed electromagnetic fields on breast cancer cell line MCF 7 using absorption spectroscopy. *Anticancer research.*.

[44] Cho H.-W., Kim S.-N., Kim K. K., Kim K., Kim K.-J. (2016). Pulsed electromagnetic fields stimulate cellular proliferation in different types of cells. *IEEE Transactions on Magnetics.*.

[45] Crocetti S., Beyer C., Schade G., Egli M., Fröhlich J., Franco-Obregón A. (2013). Low intensity and frequency pulsed electromagnetic fields selectively impair breast cancer cell viability. *PLoS One*.

The article "Evaluation of Pulsed Electromagnetic Field Effects: A Systematic Review and Meta-Analysis on Highlights of Two Decades of Research In Vitro Studies" was published in 2021. Journal: Biomed Res Int.

[46] Wójcik-Piotrowicz K., Kaszuba-Zwoinska J., Rokita E., Nowak B., Thor P. (2017). Changes in U937 cell viability induced by stress factors—possible role of calmodulin. *Journal of Physiology and Pharmacology*.

[47] Sontag W., Kalka D. (2006). No effect of pulsed electromagnetic fields on PC12 and HL-60 cells. *Radiation and environmental biophysics.*.

[48] Loja T., Stehlikova O., Palko L., Vrba K., Rampl I., Klabusay M. (2014). Influence of pulsed electromagnetic and pulsed vector magnetic potential field on the growth of tumor cells. *Electromagnetic biology and medicine.*.

[49] Sadeghipour R., Ahmadian S., Bolouri B., Pazhang Y., Shafiezadeh M. (2012). Effects of extremely low-frequency pulsed electromagnetic fields on morphological and biochemical properties of human breast carcinoma cells (T47D). *Electromagnetic biology and medicine.*.

[50] Kaivosoja E., Sariola V., Chen Y., Konttinen Y. T. (2015). The effect of pulsed electromagnetic fields and dehydroepiandrosterone on viability and osteo-induction of human mesenchymal stem cells. *Journal of tissue engineering and regenerative medicine.*.

[51] Borsje M. A., Ren Y., de Haan-Visser H. W., Kuijer R. (2010). Comparison of low-intensity pulsed ultrasound and pulsed electromagnetic field treatments on OPG and RANKL expression in human osteoblast-like cells. *The Angle Orthodontist.*.

[52] Hannay G., Leavesley D., Pearcy M. (2005). Timing of pulsed electromagnetic field stimulation does not affect the promotion of bone cell development. *Bioelectromagnetics*.

[53] Sollazzo V., Palmieri A., Pezzetti F., Massari L., Carinci F. (2010). Effects of pulsed electromagnetic fields on human osteoblastlike cells (MG-63): a pilot study. *Clinical Orthopaedics and Related Research*.

[54] Mattei M. D., Gagliano N., Moscheni C. (2005). Changes in polyamines, c-myc and c-fos gene expression in osteoblast-like cells exposed to pulsed electromagnetic fields. *Bioelectromagnetics.*.

[55] De Mattei M., Caruso A., Traina G. C., Pezzetti F., Baroni T., Sollazzo V. (1999). Correlation between pulsed electromagnetic fields exposure time and cell proliferation increase in human osteosarcoma cell lines and human normal osteoblast cells in vitro. *Bio electro magnetics*.

[56] Oladnabi M., Bagheri A., Rezaei Kanavi M., Azadmehr A., Kianmehr A. (2019). Extremely low frequency-pulsed electromagnetic fields affect proangiogenic-related gene expression in retinal pigment epithelial cells. *Iranian journal of basic medical sciences.*.

[57] Capelli E., Torrisi F., Venturini L. (2017). Low-frequency pulsed electromagnetic field is able to modulate miRNAs in an experimental cell model of Alzheimer’s disease. *Journal of healthcare engineering.*.

The article "Evaluation of Pulsed Electromagnetic Field Effects: A Systematic Review and Meta-Analysis on Highlights of Two Decades of Research In Vitro Studies" was published in 2021. Journal: Biomed Res Int.

[58] Kaszuba-Zwoińska J., Zdziłowska E., Chorobik P. (2011). Pulsing electromagnetic field and death of proliferating peripheral blood mononuclear cells from patients with acute myelogenic leukemia. *Advances in Clinical and Experimental Medicine*.

[59] Cheng Y., Qu Z., Fu X., Jiang Q., Fei J. (2017). Hydroxytyrosol contributes to cell proliferation and inhibits apoptosis in pulsed electromagnetic fields treated human umbilical vein endothelial cells in vitro. *Molecular medicine reports.*.

[60] Kubat N. J., Moffett J., Fray L. M. (2015). Effect of pulsed electromagnetic field treatment on programmed resolution of inflammation pathway markers in human cells in culture. *Journal of inflammation research.*.

[61] de Girolamo L., Viganò M., Galliera E. (2015). In vitro functional response of human tendon cells to different dosages of low-frequency pulsed electromagnetic field. *Knee Surgery, Sports Traumatology, Arthroscopy.*.

[62] Miller S. L., Coughlin D. G., Waldorff E. I., Ryaby J. T., Lotz J. C. (2016). Pulsed electromagnetic field (PEMF) treatment reduces expression of genes associated with disc degeneration in human intervertebral disc cells. *The Spine Journal.*.

[63] Okada M., Kim J. H., Hutton W. C., Yoon S. T. (2013). Upregulation of intervertebral disc-cell matrix synthesis by pulsed electromagnetic field is mediated by bone morphogenetic proteins. *Clinical Spine Surgery.*.

[64] Okada M., Kim J. H., Yoon S. T., Hutton W. C. (2013). Pulsed electromagnetic field (PEMF) plus BMP-2 upregulates intervertebral disc-cell matrix synthesis more than either BMP-2 alone or PEMF alone. *Clinical Spine Surgery.*.

[65] Guerkov H., Lohmann C., Liu Y. (2001). Pulsed electromagnetic fields increase growth factor release by nonunion cells. *Clinical Orthopaedics and Related Research*.

[66] Stolfa S., Skorvanek M., Stolfa P., Rosocha J., Vasko G., Sabo J. (2007). Effects of static magnetic field and pulsed electromagnetic field on viability of human chondrocytes in vitro. *Physiological research.*.

[67] Shah J., Midkiff P., Brandt P., Sisken B. (2001). Growth and differentiation of PC6 cells: the effects of pulsed electromagnetic fields (PEMF). *Bioelectromagnetics*.

[68] Lekhraj R., Cynamon D. E., DeLuca S. E., Taub E. S., Pilla A. A., Casper D. (2014). Pulsed electromagnetic fields potentiate neurite outgrowth in the dopaminergic MN9D cell line. *Journal of neuroscience research.*.

[69] Baranowska A., Skowron B., Nowak B. (2017). Changes in viability of rat adipose-derived stem cells isolated from abdominal/perinuclear adipose tissue stimulated with pulsed electromagnetic field. *J Physiol Pharmacol.*.

[70] Gehwolf R., Schwemberger B., Jessen M. (2019). Global responses of Il-1*β*-primed 3D tendon constructs to treatment with pulsed electromagnetic fields. *Cells.*.

The article "Evaluation of Pulsed Electromagnetic Field Effects: A Systematic Review and Meta-Analysis on Highlights of Two Decades of Research In Vitro Studies" was published in 2021. Journal: Biomed Res Int.

[71] Wu S., Yu Q., Lai A., Tian J. (2018). Pulsed electromagnetic field induces Ca^2+^-dependent osteoblastogenesis in C3H10T1/2 mesenchymal cells through the Wnt- Ca^2+^/Wnt-*β*-catenin signaling pathway. *Biochemical and biophysical research communications.*.

[72] Teven C. M., Greives M., Natale R. B. (2012). Differentiation of osteoprogenitor cells is induced by high-frequency pulsed electromagnetic fields. *Journal of Craniofacial Surgery.*.

[73] Seo N., Lee S.-H., Ju K. W. (2018). Low-frequency pulsed electromagnetic field pretreated bone marrow-derived mesenchymal stem cells promote the regeneration of crush-injured rat mental nerve. *Neural regeneration research.*.

[74] Lu T., Huang Y., Zhang C., Chai M., Zhang J. (2015). Effect of pulsed electromagnetic field therapy on the osteogenic and adipogenic differentiation of bone marrow mesenchymal stem cells. *Genet Mol Res.*.

[75] Wang J., Tang N., Xiao Q. (2015). Pulsed electromagnetic field may accelerate in vitro endochondral ossification. *Bioelectromagnetics.*.

[76] Li X., Zhang M., Bai L., Bai W., Xu W., Zhu H. (2012). Effects of 50 Hz pulsed electromagnetic fields on the growth and cell cycle arrest of mesenchymal stem cells: an in vitro study. *Electromagnetic biology and medicine.*.

[77] Meng D., Xu T., Guo F., Yin W., Peng T. (2009). The effects of high-intensity pulsed electromagnetic field on proliferation and differentiation of neural stem cells of neonatal rats in vitro. *Journal of Huazhong University of Science and Technology*.

[78] Pi Y., Liang H., Yu Q. (2019). Low-frequency pulsed electromagnetic field inhibits RANKL-induced osteoclastic differentiation in RAW264. 7 cells by scavenging reactive oxygen species. *Molecular medicine reports.*.

[79] Wang P., Liu J., Yang Y. (2017). Differential intensity-dependent effects of pulsed electromagnetic fields on RANKL-induced osteoclast formation, apoptosis, and bone resorbing ability in RAW264. 7 cells. *Bioelectromagnetics.*.

[80] Ross C. L., Harrison B. S. (2013). Effect of pulsed electromagnetic field on inflammatory pathway markers in RAW 264.7 murine macrophages. *Journal of inflammation research*.

[81] Kudo T.-a., Kanetaka H., Shimizu Y. (2013). Induction of neuritogenesis in PC12 cells by a pulsed electromagnetic field via MEK-ERK1/2 signaling. *Cell structure and function*.

[82] Vincenzi F., Targa M., Corciulo C. (2012). The anti-tumor effect of A 3 adenosine receptors is potentiated by pulsed electromagnetic fields in cultured neural cancer cells. *PLoS One.*.

[83] Solek P., Majchrowicz L., Bloniarz D., Krotoszynska E., Koziorowski M. (2017). Pulsed or continuous electromagnetic field induce p53/p21-mediated apoptotic signaling pathway in mouse spermatogenic cells _in vitro_ and thus may affect male fertility. *Toxicology.*.

The article "Evaluation of Pulsed Electromagnetic Field Effects: A Systematic Review and Meta-Analysis on Highlights of Two Decades of Research In Vitro Studies" was published in 2021. Journal: Biomed Res Int.

[84] Zou J., Chen Y., Qian J., Yang H. (2017). Effect of a low-frequency pulsed electromagnetic field on expression and secretion of IL-1*β* and TNF-*α* in nucleus pulposus cells. *Journal of International Medical Research.*.

[85] Muramatsu Y., Matsui T., Deie M., Sato K. (2017). Pulsed electromagnetic field stimulation promotes anti-cell proliferative activity in doxorubicin-treated mouse osteosarcoma cells. *In vivo*.

[86] Emes Y., Akça K., Aybar B. (2013). Low-level laser therapy vs. pulsed electromagnetic field on neonatal rat calvarial osteoblast-like cells. *Lasers in medical science.*.

[87] Wei Y., Xiaolin H., Tao S. (2008). Effects of extremely low-frequency-pulsed electromagnetic field on different-derived osteoblast-like cells. *Electromagnetic biology and medicine.*.

[88] Selvamurugan N., Kwok S., Vasilov A., Jefcoat S. C., Partridge N. C. (2007). Effects of BMP-2 and pulsed electromagnetic field (PEMF) on rat primary osteoblastic cell proliferation and gene expression. *Journal of orthopaedic research.*.

[89] Schnoke M., Midura R. J. (2007). Pulsed electromagnetic fields rapidly modulate intracellular signaling events in osteoblastic cells: comparison to parathyroid hormone and insulin. *Journal of orthopaedic research.*.

[90] Chang W. H. S., Chen L. T., Sun J. S., Lin F. H. (2004). Effect of pulse-burst electromagnetic field stimulation on osteoblast cell activities. *Bioelectromagnetics*.

[91] Miyamoto H., Sawaji Y., Iwaki T. (2019). Intermittent pulsed electromagnetic field stimulation activates the mTOR pathway and stimulates the proliferation of osteoblast-like cells. *Bioelectromagnetics.*.

[92] Suryani L., Too J. H., Hassanbhai A. M. (2019). Effects of electromagnetic field on proliferation, differentiation, and mineralization of MC3T3 cells. *Tissue Engineering Part C: Methods.*.

[93] Li K., Hui Y., Ma S. (2011). Inhibition of bone formation by high intensity pulsed electromagnetic field in MC3T3-E1 cells. *Progress in electromagnetics research.*.

[94] Diniz P., Shomura K., Soejima K., Ito G. (2002). Effects of pulsed electromagnetic field (PEMF) stimulation on bone tissue like formation are dependent on the maturation stages of the osteoblasts. *Bio electro magnetics*.

[95] Patterson T. E., Sakai Y., Grabiner M. D. (2006). Exposure of murine cells to pulsed electromagnetic fields rapidly activates the mTOR signaling pathway. *Bioelectromagnetics*.

[96] Xu H., Zhang J., Lei Y. (2016). Low frequency pulsed electromagnetic field promotes C2C12 myoblasts proliferation via activation of MAPK/ERK pathway. *Biochemical and biophysical research communications.*.

The article "Evaluation of Pulsed Electromagnetic Field Effects: A Systematic Review and Meta-Analysis on Highlights of Two Decades of Research In Vitro Studies" was published in 2021. Journal: Biomed Res Int.

[97] Choi J., Shin S., Kim S. (2010). In vitrostimulation with a strongly pulsed electromagnetic field on rat basophilic leukemia cells. *Journal of Applied Physics*.

[98] Chen J., He H.-C., Xia Q.-J., Huang L.-Q., Hu Y.-J., He C. Q. (2010). Effects of pulsed electromagnetic fields on the mRNA expression of RANK and CAII in ovariectomized rat osteoclast-like cell. *Connective tissue research.*.

[99] Tang X., Coughlin D., Ballatori A. (2019). Pulsed electromagnetic fields reduce interleukin-6 expression in intervertebral disc cells via nuclear factor-*κβ* and mitogen-activated protein kinase p 38 pathways. *Spine.*.

[100] Kavand H., Haghighipour N., Zeynali B., Seyedjafari E., Abdemami B. (2016). Extremely low frequency electromagnetic field in mesenchymal stem cells gene regulation: chondrogenic markers evaluation. *Artificial Organs.*.

[101] Lohmann C., Schwartz Z., Liu Y. (2003). Pulsed electromagnetic fields affect phenotype and connexin 43 protein expression in MLO-Y4 osteocyte-like cells and ROS 17/2.8 osteoblast-like cells. *Journal of orthopaedic research.*.

